The article "Updated Pharmacological Effects of Total Phenolic Acid on the Meningeal Microcirculation in Mice" was retracted in 2023. Reasons: signs of a paper mill; suspected computer-generated content; unreliable results or conclusions; lack of ethics approval or compliance.

# Updated Pharmacological Effects of Total Phenolic Acid on the Meningeal Microcirculation in Mice

**DOI:** 10.1155/2022/8441050

**Published:** 2022-03-26

**Authors:** Hui Zhao, Jiaojiao Jia, Ming Bai, Mingsan Miao

**Affiliations:** ^1^Department of Pharmacology, School of Pharmacy, Chengdu University of Traditional Chinese Medicine, Chengdu 611137, China; ^2^College of Postgraduates, Henan University of Chinese Medicine, Zhengzhou 450000, China

## Abstract

**Objective:**

To investigate the effects of total phenolic acid on meningeal microcirculation in mice.

**Methods:**

A total of 84 healthy mice were randomly divided into the blank group, the model group, the positive control Western medicine group, the positive control Chinese medicine group, and the large, medium, and small doses of the total phenolic acid group, with 12 rats in each group. The corresponding drug was given to the group once a day for one week, and the litter was changed at 9 : 00 on the 6th day, and the water fasted. On the 7th day, the groups continued to be administered and weighed. After 1 h, the percentage of decrease in the perfusion of the mice was measured.

**Results:**

Compared with the blank group, the percentage of perfusion decreased significantly in the model group, indicating that the model was successful. Compared with the model group, the nimodipine group, the Naoluotong group, and the high-dose succulent total phenolic acid group were perfused. The percentage of decrease was significantly decreased (*P* < 0.01), and the percentage of perfusion decreased in the middle and small doses of the total phenolic acid group (*P* < 0.05), indicating that the percentage of mice perfused decreased by the administration of each group.

**Conclusion:**

Total phenolic acid can reduce the percentage of mean perfusion of microcirculation in animals and reduce brain damage.

## 1. Introduction

The big blood vine is the dried cane and root of the big vine, *Sargentodoxa cuneata* (Oliv) Rehd.et Wils. The big blood vine is flat and bitter and enters the large intestine and liver [1]. Chinese medicine believes that *S. sinensis* has the effects of detoxification, heat-clearing, Qi and blood circulation, phlegm and blood stasis, swelling and dispersing, relieving pain, passing through, and poisoning. Therefore, it is clinically used to treat appendicitis, irregular menstruation, uterine bleeding, intestinal fistula, abdominal pain, amenorrhea, amenorrhea, rheumatism, pain, bruises, etc. [2]. So far, many active ingredients have been isolated from the *Spatholobus*, mainly compounds such as quinones, phenols, and flavonoids. Chemical studies have shown that phenolic acids in the *Spatholobus* have unique physiological and pharmacological activities. This study aimed to investigate the effects of total phenolic acids on meningeal microcirculation in mice [3].

## 2. Experimental Materials

### 2.1. Experimental Animals

Kunming mice, 84 males, SPF grade, weight 18–22 g, provided by: Shandong Lukang Pharmaceutical Co., Ltd. (certificate no.: 37005400000009). Laboratory certificate number SYXK (Yu) 2015–0005.

### 2.2. Drugs and Reagents

Total phenolic acid, *Daphne sinensis*, provided by Analytical Chemistry Laboratory, Henan University of Traditional Chinese Medicine, 70.04%; nimodipine (positive control Western medicine), Yabao Pharmaceutical Group Co., Ltd., batch number 140861; Naoluotong Capsule (positive control Chinese medicine), Jilin Jinbao Pharmaceutical Co., Ltd. production, batch number 150401; pentobarbital sodium, Shanghai Xinya Pharmaceutical Co., Ltd., batch number 921019; saline, Henan Kelun Pharmaceutical Co., Ltd., batch number C117112904-1; medical ethanol (alcohol), Xinxiang Sanwei Disinfection Preparation Co., Ltd., batch number 20180605.

### 2.3. Experimental Instruments

Electronic balance, Shanghai Precision Scientific Instrument Co., Ltd. (FA2204B), and speckle full-frame real-time scanning imager, PeriCam PSI were used in this study.

## 3. Experimental Methods

### 3.1. Grouping

84 healthy male mice with SPF grade and bodyweight of 18 g–22 g were normally reared for 3 days, weighed, and randomly divided into blank group, model group, positive-control Western medicine group, positive-control Chinese medicine group, large, medium, and small doses. Group 7 consists of blood vine total phenolic acid group, 12 mice per group.

### 3.2. Modeling Methods and Administration

The study groups were nimodipine group (positive control Western medicine, the dose is 15 times of clinical dosage, 30 mg/kg), naoluotong group (medical medicine in the positive control, the dosage is 15 times of clinical dosage, 750 mg/kg), large, medium, and small doses of the total phenolic acid group (450 mg/kg, 225 mg/kg, 112.5 mg/kg, respectively, 30 times, 15 times, and 7.5 times the dose of clinical human body), blank group, and model group. The same volume of normal saline was administered (the volume of each group was 0.1 ml/5 g). The corresponding drug was administered once a day for one week, the litter was changed at 9 : 00 pm on the sixth day, and the water fasted. The body weight of each mouse was measured before the last administration, and the percentage of decrease in the perfusion amount of the mice was measured 1 hour after the administration.

### 3.3. Detection Indicators and Detection Methods

The computer and accessory equipment needed for the measurement and the Perimed instrument were turned on. The instrument was left for 5 minutes before using the instrument to warm up the instrument. The LED indicator was observed for stopping of flashing and indication that the detection process can be performed. The PIMsoft software was opened, and the PeriCam PSI system was entered. The conditions and modes required for the experiment were adjusted, the operating distance was adjusted to 10 cm, the height and width of the experimental test were adjusted to 2 cm, the sampling frequency was set to 23 pictures/s, the step length was set to medium, the duration was set to stop at the end, all data settings were made sure to be successful, and the experiment operation was started by clicking OK [4].

Half an hour after the last administration, the mice were anesthetized (0.03 ml/10 g) with 3% pentobarbital sodium, and the mice were fixed in a prone position using a rat plate. During the operation, the skin of the mouse skull was cut open, and the hemostatic forceps were pulled apart along the incision. The cotton wool containing the H_2_O_2_ solution was gently used to wipe the mouse skull, and the muscle tissue entrained on the skull surface was peeled off with a marker. The mouse coronal wind and the sagittal suture of the brain are marked. During the operation, the mouse is placed within the recommended distance of the instrument, and the control instrument is parallel to the mouse monitoring brain point, and the beam can be illuminated at the mark. It is perpendicular to the detection point. After setting the instrument distance to the optimal distance of the operation and selecting the experimental scan area range, the “Record” button was clicked to start the recording and monitoring of the mouse perfusion volume, and the blood perfusion volume of the mouse was measured within 2 min after the operation is completed and stabilized.

After the above operation was completed, the mice were released and the mice were again fixed in the supine position with the rat plate, and the bilateral common carotid arteries were separated and ligated (the blank group only separated the bilateral common carotid arteries without ligating the common carotid artery), and the recording was small. The blood perfusion of mice was measured within 2 mins after stabilization [5].

The mean blood perfusion amount was taken from 1 min 50 s to 2 min as the average perfusion amount before ligation, and the average blood perfusion amount in the period of 3 min 50 s to 4 min was taken as the average perfusion amount after ligation. After all surgical procedures have been completed, the experimental report is exported and the data analyzed.

### 3.4. Statistical Methods

Data analysis was performed using the SPSS 19.0 statistical software package for statistical processing of the data. The measurement data were expressed as mean ± standard deviation $\left(\bar{X}\pm s\right)$. One-way ANOVA was used for comparison between groups, and the least significant difference was used for the variance test. In the LSD method, the variance is tested by the Games–Howell method, and the grade data are verified by the Radit test.

## 4. Experimental Results

### 4.1. Effects on Meningeal Microcirculation before and after Carotid Artery Ligation in Mice

It can be seen from Table 1 that compared with the blank group, the percentage of the decrease in the perfusion volume of the model group increased significantly, indicating that the model was successful; compared with the model group, the positive control western medicine group, the positive control traditional Chinese medicine group, and the high-dose total phenolic acid of Daxueteng can alleviate the symptoms of lack of perfusion. The percentage of perfusion decreased significantly in the acid group (*P* < 0.01) (Figures 1–4), and the percentage of perfusion in the middle and small doses of the total phenolic acid group was significantly decreased (*P* < 0.05) (Figures 5–7), indicating that the administration of each group can be reduced [6, 7]. The percentage of rat perfusion decreased. The experimental data suggest that the effect of phenolic acid on meningeal microcirculation in cerebral ischemia mice is observed in a dose-dependent manner. 450 mg/kg total phenolic acid is used to improve the model of cerebral ischemia. Mouse meningeal microcirculation has a good preventive effect.

### 4.2. Changes in the Meningeal Microcirculation Perfusion

The changes in the meningeal microcirculation perfusion are shown in Figures 1–7.

## 5. Conclusions

Cerebral ischemia is a common clinical disease with a high mortality rate, second only to cancer and myocardial infarction [8]. Cerebral ischemia is caused by a severe lack of blood flow in the brain during the preonset period. According to the survey results of cardiovascular and cerebrovascular diseases in recent years, the number of cerebrovascular diseases has increased year by year [9]. The blood supply disorder in the brain causes the oxygen content in the brain tissue to decrease, and the lack of oxygen supply to the blood vessels leads to abnormal metabolism of the tissues and organs of the body, which will lead to abnormal morphological changes. The most obvious pathological response to ischemic cerebral ischemia is neuronal necrosis or apoptosis. TCM syndrome differentiation and treatment believe that the cause of cerebral ischemia is due to Qi deficiency, poor blood flow, brain loss, lack of liver and kidney Yin, Qi stagnation, Qi turbidity, etc. [10]. Therefore, Chinese medicine often uses Qi and blood, phlegm and blood stasis, phlegm and blood stasis, warming liver and kidney, clearing heat and nourishing Yin to treat patients with cerebral ischemia [11, 12].

The body microcirculation system can directly participate in the information, substance, and energy transfer between various tissues and cells, and judge the occurrence and development of diseases by detecting the flow state of blood, lymph, and tissue fluid [13]. It is considered that the application of microcirculation technology is excellent for disease progression. Prompt role. With the advancement of microcirculation testing instruments and methods of use as well as the continuous specification of observation indicators and operating procedures, the application of drug clinical research has gradually increased and has become an important technology platform for obtaining innovative results [14]. Dynamic visualization microcirculation technology is a process of organically merging imaging and information technology, and observing the state of microcirculation through fluorescent labeling. The technique of replacing the resting image with dynamic visual graphics, this technology provides new technical support for studying the mechanism of promoting blood circulation and removing blood stasis drugs to improve microcirculation [15].

The gold index of cerebral ischemia is reflected in the change of perfusion volume. A significant decrease in perfusion volume indicates successful model replication. The effect of total phenolic acid on the percentage of perfusion decreased before and after bilateral common carotid artery ligation in mice, suggesting that total phenolic acid can reduce the percentage of mean microcirculation perfusion of animals and reduce brain damage to large doses. The total phenolic acid group is the best. Therefore, it can be proved that Daxue can improve the microcirculation disturbance caused by cerebral ischemia by promoting blood circulation, clearing away heat and detoxification, providing the clinical basis for Chinese medicine treatment of cerebral ischemic diseases, and bringing social benefits and economic benefits [16].

## Figures and Tables

**Figure 1:** Blank group.

**Figure 2:** Model group.

**Figure 3:** Positive-control Western medicine group.

**Figure 4:** Positive-control Chinese medicine group.

**Figure 5:** Large dose of big blood vine total.

**Figure 6:** Medium dose of big blood vine total phenolic acid group.

**Figure 7:** Low dose of big blood vine total phenolic acid group.

**Table 1:** Effect of meningeal microcirculation before and after carotid artery ligation in mice $\left(\bar{X}\pm s\right)$.

Group	Number of animals	Dose (mg/kg)	Percentage of perfusion reduction (%)
Blank group	12	—	4.74 ± 0.89^*∗∗*^
Model group	12	—	33.03 ± 4.48
Positive control western medicine group	12	30	23.06 ± 4.51^*∗∗*^
Positive control Chinese medicine group	12	750	21.10 ± 4.92^*∗∗*^
Large dose of big blood vine total phenolic acid group	12	450	24.14 ± 5.00^*∗∗*^
Medium dose of big blood vine total phenolic acid group	12	225	28.23 ± 4.70^*∗*^
Low dose of big blood vine total phenolic acid group	12	112.5	29.23 ± 5.49^*∗*^

Compared with the model group, ^∗∗^*P* < 0.01, ^∗^*P* < 0.05.

## Data Availability

The datasets used and/or analyzed during the current study are available from the corresponding author on reasonable request.
